This article has been retracted.

# Intraosseous Calcaneal Lipoma Misdiagnosed as Plantar Fasciitis: An Orthopedic Case From Family Practice

**DOI:** 10.7759/cureus.21136

**Published:** 2022-01-11

**Authors:** Alaa M Alnooh, Bashayer F Al Furaikh, Abdullah M Alaithan, Abdulaziz K Halawani, Mohammed F Al-Khalifah, Mohammad O Abu Zahirah, Mutasim H Alhasani, Abdullmgeed A Asiri, Aqeel H Alrashid, Eyad H Alfaqih, Mohammed A Khair, Seddiqa S Naiser, Yaqeen S Alkamel, Abdulaziz A Al Mohammed, Faisal Al-Hawaj

**Affiliations:** 1 College of Medicine, Alfaisal University, Riyadh, SAU; 2 College of Medicine, King Faisal University, Hofuf, SAU; 3 General Practice, King Abdullah Medical City, Riyadh, SAU; 4 College of Medicine, Umm Al-Qura University, Mecca, SAU; 5 College of Medicine, King Saud University, Riyadh, SAU; 6 College of Medicine, King Khalid University, Abha, SAU; 7 College of Medicine, Taif University, Taif, SAU; 8 College of Medicine, King Saud Bin Abdulaziz University For Health Sciences, Riyadh, SAU; 9 College of Medicine, Xi’an Jiaotong University, Xi'an, CHN; 10 College of Medicine, Imam Abdulrahman Bin Faisal University, Dammam, SAU

**Keywords:** lipoma, plantar fasciitis, heel pain, intraosseous, case report

## Abstract

Foot pain is a prevalent musculoskeletal complaint with plantar fasciitis being one of the most common underlying etiologies. Diagnostic imaging studies are rarely performed for patients with plantar fasciitis. We report the case of a 34-year-old woman with a six-month history of left heel pain that was worsened by prolonged standing and walking. She was diagnosed as having plantar fasciitis. Considering the lack of clinical improvement on conservative measures, the patient underwent a plain radiograph, which demonstrated a geographic radiolucent lesion in the calcaneus with well-defined non-sclerotic margins. Subsequently, a computed tomography scan re-demonstrated the lesion as having a fat-attenuation appearance that was classic of lipoma. The patient underwent surgical excision of the tumor and the histopathological examination of the specimen revealed spindle cell lipoma. The patient had complete resolution of the pain following the surgery. Intraosseous lipoma is a very rare benign primary bone tumor. The case demonstrated that the intraosseous lipoma may have similar clinical features to plantar fasciitis. Hence, physicians should keep a high index of suspicion for the alternate diagnoses of plantar fasciitis in patients who do not exhibit any clinical improvement despite a prolonged period of conservative management.

## Introduction

Musculoskeletal complaints are very common and are one of the most frequent reasons for general practice visits. It is estimated that up to one-third of visits to primary care centers are related to musculoskeletal disorders [1]. Heel pain develops in up to 10% of people above the age of 50 years [2]. Many factors have been associated with hindfoot and heel pain which are usually related to mechanical factors. The common causes of chronic heel pain include plantar fasciitis, tarsal tunnel syndrome, sinus tarsi syndrome, and subtalar arthritis. Plantar fasciitis affects over a million individuals in the United States every year. The clinical diagnosis of plantar fasciitis is based on the clinical features and diagnostic imaging is seldom requested. The management of plantar fasciitis is primarily conservative. However, the management of plantar fasciitis can be challenging and refractory to conservative treatment [3]. Here, we report the case of a young patient with chronic heel pain that was initially diagnosed as having plantar fasciitis and eventually found to have intraosseous spindle cell lipoma, a rare benign bone neoplasm.

## Case presentation

A 34-year-old woman presented to the family and community medicine clinic with a complaint of left heel pain for six months duration. She described the pain as sharp in nature. The pain had gradual onset and it had been increasing in severity. The pain was aggravated by standing or walking for a prolonged period. The pain was not associated with a history of sensory or motor weakness. She did not have any pain in the right foot. The patient reported no history of trauma-related to her pain. There was no history of morning stiffness in her heels. The patient did not complain of any joint pain, skin rash, or muscle weakness, fever, or weight loss.

The patient visited multiple orthopedic clinics previously. She was diagnosed as having plantar fasciitis. The condition was attributed to her obesity. The impact of obesity on plantar fasciitis was discussed. She was advised to undergo lifestyle modification to reduce her weight. She was offered symptomatic treatment with non-steroidal anti-inflammatory medications. However, these analgesics gave no significant improvement. She also underwent several sessions of physiotherapy with stretching exercise therapy.

The past medical history was remarkable for polycystic ovarian syndrome for which she was taking metformin 500 mg daily. No history of previous surgical intervention. The patient was a non-smoker and had no history of alcohol consumption. She worked as a computer science professor. No history of rheumatological diseases in the family.

Upon examination, the patient was obese and had a body mass index of 37.2 kg/m2. There was no tenderness over the heel. No evidence of soft tissue inflammation in the left foot. Laboratory investigations revealed normal hematological and biochemical parameters. Autoimmune antibodies panels, including antinuclear antibody, anti-dsDNA, anti-Smith, anti-Ro, and anti-La, were negative.

Considering the chronicity of the pain and unresponsiveness to non-surgical treatments, the patient underwent a plain radiograph for the ankle and heel. The radiograph demonstrated a geographic radiolucent lesion in the anterior part of the calcaneus with well-defined non-sclerotic margins (Figure 1). The radiological differential diagnoses for this lesion were broad and included fibrous dysplasia, aneurysmal bone cyst, enchondroma, lipoma, and osteomyelitis. In order to narrow the diagnosis, a computed tomography scan of the foot was performed. The scan re-demonstrated the intraosseous lesion as having a fat-attenuation appearance that was classic of lipoma (Figure 2).

**Figure 1:** Plain radiograph of left ankle showing a radiolucent lesion (arrow) in the calcaneum with well-defined margins.

**Figure 2:** Coronal (A) and axial (B) CT images show well-defined calcaneal lesion (arrow) with a fat density.

Subsequently, the patient underwent surgical intervention and the tissue on the target area was removed and replaced by bone grafting. Histopathological examination of the lesion showed mature adipose cells with interposed uniform spindle cells conferring the diagnosis of spindle cell lipoma (Figure 3). The patient was discharged on the fourth postoperative day. Due to the coronavirus disease 2019 pandemic, the follow-up was made with virtual clinics. She was followed up for three months and had no recurrence of her chronic pain.

**Figure 3:** Histopathological image shows mature adipose cells with interposed uniform spindle cells.

## Discussion

We reported a rare case of osseous lipoma of the calcaneus presenting with chronic heel pain that was mistakenly diagnosed as plantar fasciitis. Intraosseous lipoma is a very rare benign bone tumor accounting for less than 1 per 1000 of all primary bone tumors [4]. Such tumors may develop at any age and have no gender predilection. Intraosseous lipoma tends to have non-specific clinical manifestations and it is often misdiagnosed, as in our case [5]. It may be misdiagnosed as plantar fasciitis, plantar bursitis, stress fracture, aneurysmal bone cyst, and other benign tumors. However, the vast majority of intraosseous lipoma cases are asymptomatic and are detected incidentally on imaging [6].

The pathogenesis of intraosseous lipoma remains unclear. It is believed that intraosseous lipoma is a true benign neoplasm of the yellow marrow of the bone. However, other hypotheses suggest that intraosseous lipoma arises from fat metaplasia from previous trauma or infection [6]. Spindle cell lipoma is a distinct variant of lipoma that accounts for less than 1.5% of all lipomas [7]. In contrast to the typical lipoma, spindle cell lipoma has male predilection which might be due to the presence of androgen receptors in the tumor cells of spindle cell lipoma [7].

Imaging studies can make the diagnosis of intraosseous lipoma with high accuracy. Radiographs show a lucent intramedullary lesion that may be surrounded by a thin sclerotic rim. The lesion may have central calcification and mild cortical expansion [6]. A computed tomography scan demonstrates an intraosseous lesion of fat density that may have evidence of bone remodeling. It is worth noting that Milgram et al. [8] have proposed a staging system for intraosseous lipoma. The first stage of intraosseous lipoma has viable fat cells. The second stage is considered a transitional stage and composed of both viable and necrotic adipose tissue and calcification. The third stage includes necrotic fat and calcification with reactive bone changes. The magnetic resonance imaging findings depend largely on the stage of the lipoma [8]. In the early stages of the intraosseous lipoma, the magnetic resonance imaging shows a high signal intensity in T1 and T2-weighted images that are isointense to the subcutaneous fat and demonstrates suppression on the short tau inversion recovery sequence [9]. However, later stages of lipoma may have areas of low signal intensity in T1 and high signal intensity in T2 representing fat necrosis or cyst formation along with signal void areas in keeping with calcification [5]. In the present case, magnetic resonance imaging was noted performed because of its cost.

## Conclusions

Intraosseous lipoma is a very rare benign primary bone tumor. The case demonstrated that the intraosseous lipoma may have similar clinical features to plantar fasciitis. Hence, physicians should keep a high index of suspicion for the alternate diagnoses of plantar fasciitis in patients who do not exhibit any clinical improvement despite a prolonged period of conservative management. Surgical excision of the tumor is curative and results in complete resolution of the pain.
